The article "Modular Furniture Design by Using Intelligent Platform and Wireless Sensors" was published in 2022. Journal: Comput Intell Neurosci.

# Modular Furniture Design by Using Intelligent Platform and Wireless Sensors

**DOI:** 10.1155/2022/2586711

**Published:** 2022-11-23

**Authors:** Wu Shilin

**Affiliations:** School of Fine Arts & Design, Guangzhou University, Guangzhou, Guangdong 510006, China

## Abstract

The continuous development of the society has led to the improvement of people's quality of life and consumption level. At the same time, peoples demand for all aspects of production and life is also increasing, thus promoting the emergence and innovation of intelligent household appliances. To manage these devices conveniently and quickly and enrich family life, “smart home” bureau plays a very important role. Smart home, which enters people's family life, uses communication technology, Internet connection technology, automatic fire control technology, network wiring technology, and visual and audio transmission technology to communicate with home. Mobile terminals have been developed, and more and more PC functions have been realized. Based on the hardware platform of the smart home management system, two solutions were put forward. The first solution is combined with the current 5G network, and through it, the user can control the mobile phone and other mobile terminals on the corresponding application operation instructions to create. The second solution is the design of the web server intelligent management system, for relevant information. It is collected into the database of the server, allows remote access to the node and subscriber information related to storage in the database through the Internet, and searches the information to control the home lighting and temperature. This system is designed to imitate the modular scheme, which includes the central control module, sensor data acquisition module, and software module. Finally, on the browser side and the electronic devices of Android operating system, it realizes the wireless control of lighting, air conditioning, washing machine, and other devices, as well as the detection of the home environment.

## 1. Introduction

Smart home, on the surface, means to make the home smart; in fact, it is to add smart modules in the home to make people's lives more convenient and better. This term has been very popular in China in recent years. In fact, as early as the twentieth century, in 1984, smart buildings were first built and then Western countries started systematic smart home research. With the continuous development of science and technology, the level of fine electronic technology and computer technology has also been promoted to a great extent. People's demand for intelligence in various scenes of work, family, and social life is also becoming higher. The continuous development of the industry has also brought about dual innovation in concept and application. In 1999, the concept of intelligent management of power equipment, such as the Internet of things, was first proposed. This concept and the application have been introduced into the ranks of high-frequency technology. With recent technological developments and breakthroughs, more and more wireless communications, sensor technology, and some smarter sensing technologies have been applied to the Internet of Things. The concept of the Internet of Things has far exceeded current expectations. The smart home system based on the Internet of Things is a technology that integrates electronics, communications, sensors, cloud computing, and other disciplines to improve living standards. With the popularization of Internet of Things technology, various manufacturers have introduced their own smart home systems and adopted a variety of communication methods. The data acquired by the home center controller (coordinator) from each sensor are sent to a mobile terminal, such as a mobile phone in real-time, via an application on the mobile terminal of the home gateway to take countermeasures and monitor and process at the home.

## 2. Related Works

At present, the intelligent home network control system has three solutions of PC architecture and MCU architecture embedded architecture. To be able to remotely confirm the working status of each device in the home and perform remote operation, it is hoped that the internal network composed of household devices can be connected to some public communication platforms such as the Internet, GSM/GPRS, 3G mobile network, etc. [1]. Literature introduced the realization of a smart gateway to a smart home system [2]. As the internal network connects home equipment and the external public network, the smart gateway as the core unit of the smart home system is the top priority in the research of smart home. ResidentialGatewayGroup (RG) is the first company that represents the use of the centralized intelligent interface of the home smart gateway. RG connects the home network with the home external network [3]. The home gateway is defined as a simple, standardized, intelligent, and flexible interface device, which can receive information from various external networks and send it to a device on the home network. Cisco Systems defines the home gateway as an intelligent gateway between the network information equipment and the home intelligent broadband access network. Literature Home Gateway enables simultaneous access between “WAN” and “LAN” [4]. This enables the home gateway to be integrated into the “WAN” and “u” (broadband) networks. Literature smart gateways are the physical and logical core of smart home networks. However, it is difficult to unify the current standards of home gateways [5]. Cooperation between smart community developers and property management companies is still difficult to achieve. Many smart home manufacturers have established their own smart gateways. In recent years, China's housing construction industry has developed rapidly. To realize the intelligence of daily life, high-tech electronic information technology has become a top priority. Smart home is a perfect combination of modern high technology, modern architecture, and modern life concepts [6]. Speeding up the development of smart homes will greatly promote the development of science and technology in the country. Literature believes that the smart gateway is the core unit of the smart home system [7]. The successful development of the smart gateway will greatly improve the technical content of the residence. Literature promotes the development of the country's housing construction industry [8]. The research goal of this paper is to design and develop a small smart home control system with perfect functions, low cost, and convenient construction and installation. Based on the iovt2-2530 hardware platform, design, and research, the central control software for the system series information management platform is through the Android platform. The smart home control system can be installed through mobile phones and other terminals to remotely control the home and obtain information about various parts of the house [9]. The terminal can always know the temperature, humidity, power consumption, pressure of the water pipe, and safety information of the house, and the user can control each node through the terminal and take appropriate measures based on the main control information.

## 3. Optimized Design of Modular Home Based on Artificial Intelligence

### 3.1. Design Method of Optimized Function

The above content discusses the monitoring functions of smart products. However, the ultimate goal is an independent task. WSN alone is not enough to monitor smart products and control the automatic adjustment of fuzzy PID. On this basis, it is necessary to realize the two main functions of “optimization” and “voluntary” [10]. Optimization is the improvement of intelligent product performance and troubleshooting, such as autonomous operation, including cooperation with other products and systems, self-help enhancement of product performance, self-diagnosis, and self-service of faults. Therefore, in this chapter, we will design intelligent product optimization and autonomous functions and enable algorithms to achieve optimization functions by monitoring data and control functions. The design can be improved by evaluating the maturity of the optimization function through the number of triangular fuzzy. The three functions of fusion rate monitoring, control, and optimization are used to realize the independent function of intelligent products, and after the evaluation of the triangular fuzzy quantity has been mature, the design of the independent function is determined.

Optimization is the third function of smart products. After monitoring data and control functions, ILCS is used to improve the performance of smart products and implement fault diagnosis. The design process of the intelligent product optimization function is shown in the figure. Iterative learning includes non-linear control and control input distortion. If the interference state and the desired trajectory of the output are determined, the trailing desired trajectory will be determined [11]. If the variables of the learning rule of the selection loop PD are mastered, the state variables and output variables will be in a specific time zone, and the iterative learning control algorithm will converge. For optimization features, a number of triangle blurs to assess maturity and improve the design is used. The optimization function of smart products is based on the monitoring function and is realized through multiple iterations of the control algorithm. When smart products are running, performance is not always the best. ILCS seeks appropriate control input and makes the actual performance of smart products closer to the best performance within time, so as to achieve the goal of optimization [12]. The first step is to give the expected track *y*_*d*_(*t*) of the smart product, select the initial control input *u*_0_(*t*) in two steps, namely the initial interference state *w*_0_(*t*) and the initial interference output v0(*t*), and confirm the state of the smart phone product *x*_0_ (zero) and initial execution output *y*_0_ (zero) using three inputs *u*_0_(*t*), interference state *w*_0_(*t*), and interference output *v*_0_(*t*) control program intelligent application products and actual output error *y*_0_(*t*) *E*_0_ (*t*) = *y*_*d*_ (*t*) ∼ *y*_0_ step (*t*); after iterative learning, the next control input is the fifth step of *u*_1_(*t*), the output error is ILCS traditional feedback control, and steps 2, 3, and 4 are repeated until you use more information than the system. ILCS uses more information than traditional feedback control systems. ILCS uses the control input of the current operation at the same time. For *u*_*k*_(*t*) and the control input *u*_*k*_−1(*t*) of the last operation, the conventional feedback control system only uses the control input *u*_*k*_(*t*) of the current operation. The control input *u*_*k*_(*t*) can be calculated offline or online. Similarly, the new control input *u*_*k*_ +1(*t*) in the memory will refresh the old control input *u*_*k*_(*t*).

(1) $$\begin{array}{c} \begin{array}{c} x_{k}^{\prime }\left(t\right)=f\left(x_{k}\left(t\right),t\right)+Bu_{k}\left(t-\theta \right)+\omega_{k}\left(t\right)\text{,}\\ y_{k}\left(t\right)=Cx_{k}\left(t\right)+v_{k}\left(t\right)\text{.} \end{array} \end{array}$$

However, *t* ∈ [0,], *K* is the number of repetitions, UK(*T*) ∈ RP, XK(*T*) ∈ RM, and YK(*T*) ∈ RN are the control input, state, and output of the system, respectively, wk(*T*) ∈ . RM and VK(*T*) ∈ RN are state disturbances and output disturbances, respectively. As shown in the figure, when wk (*T*) = 0 and VK (*T*) = 0, any bounded expected trajectory YD is assumed to be state XD (*T*) and initial state XD (0) only from bounded control inputs UD (*T*) and (*T*).

(2) $$\begin{array}{c} x_{d}^{\prime }\left(t\right)=f\left(x_{d}\left(t\right),t\right)+Bu_{d}\left(t-\theta \right)\text{,}\\ y_{d}\left(t\right)=Cx_{k}\left(t\right)\text{.} \end{array}$$

**Hypothesis 1 .**

there are nonnegative real numbers “1, 2, 3”. For any *k* > 0 and *t* ∈ [0, 2], it satisfies the nonnegative real numbers “1”, “2” and “(0) (0)” ≤ “3” of any *k* > 0 and *t* ∈ [0]. Suppose 3: for any *x*_1_ (*T*), *x*_2_(*T*) ∈ r m, the non-linear function *f* () satisfies the Lipschitz condition.

(3) $$\begin{array}{c} \left\|f\left(x_{1}\left(t\right),t\right)-f\left(x_{2}\left(t\right),t\right)\right\|\leq L_{f}\left\|x_{1}\left(t\right)-x_{2}\left(t\right)\right\|\text{,} \end{array}$$

where *L*_*f*_ is Lipschitz constant. The ILCS of smart products adopts PD-type learning law:

(4) $$\begin{array}{c} u_{k+1}\left(t\right)=u_{k}\left(t\right)+\Gamma \left[e_{k}^{\prime }\left(t+\theta \right)+Le_{k}\left(t+\theta \right)\right]\text{,}\left\|I-\Gamma CB\right\|\leq p\leq 1\text{,}\Delta u_{k+1}\left(t\right)=u_{d}\left(t\right)-u_{k+1}\left(t\right)=\Delta u_{k}\left(t\right)-\Gamma \left(e_{k}^{\prime }\left(t+\theta \right)+Le_{k}\left(t+\theta \right)\right)=\left(I-\Gamma CB\right)\Delta u_{k}\left(t\right)-\Gamma C\left[f\left(x_{d}\left(t+\theta \right)-f\left(x_{k}\left(t+\theta \right)\right)\right)\right]-\Gamma LC\Delta x_{k}\left(t+\theta \right)+\Gamma C\omega_{k}\left(t+\theta \right)+\Gamma \left(I+L\right)v_{k}\left(t+\theta \right),\left\|\Delta u_{k+1}\left(t\right)\right\|,\leq \left\|I-\Gamma CB\right\|\left\|\Delta u_{k}\left(t\right)\right\|+\Gamma \left(L_{f}I+L\right)C\left\|\Delta x_{k}\left(t+\theta \right)\right\|+\Gamma C\varepsilon_{1}+\Gamma \left(I+L\right)\varepsilon_{2}x_{k}\left(t+\theta \right)=x_{k}\left(0\right)+\int_{-\theta }^{t-\theta }\left[f\left(x_{k}\left(\tau +\theta \right)\right)+Bu_{k}\left(\tau \right)+\omega_{k}\left(\tau +\theta \right)\right]d\tau ,x_{d}\left(t+\theta \right)=x_{d}\left(0\right)+\int_{-\theta }^{t-\theta }\left[f\left(x_{d}\left(\tau +\theta \right)\right)+Bu_{d}\left(\tau \right)\right]d\tau \Delta x_{k}\left(t+\theta \right)=\left[x_{d}\left(0\right)-x_{k}\left(0\right)\right]+\int_{-\theta }^{\tau -\theta }\left[f\left(x_{d}\left(\tau +\theta \right)\right)-f\left(x_{k}\left(\tau +\theta \right)\right)+B\Delta u_{k}\left(\tau \right)-\omega_{k}\left(\tau +\theta \right)\right]d\tau ,\left\|\Delta u_{k+1}\left(t\right)\right\|\leq \left\|I-\Gamma CB\right\|\left\|\Delta u_{k}\left(t\right)\right\|+\Gamma \left(L_{f}I+L\right)CB\int_{-\theta }^{\tau -\theta }e^{L_{f}\left(t-\tau \right)}\left\|\Delta u_{k}\left(\tau \right)\right\|d\tau +\Gamma \left[\left(L_{f}+1\right)I+L\right]C\varepsilon_{1}+\Gamma \left(I+L\right)\varepsilon_{2}+\Gamma \left(L_{f}I+L\right)C\varepsilon_{3,}\left\|\Delta u_{k+1}\left(t\right)\right\|\leq \left\|I-\Gamma CB\right\|\left\|\Delta u_{k}\left(t\right)\right\|+\Gamma \left(L_{f}I+L\right)CB\left\|h\left(t\right)\right\|+\Gamma \left[\left(L_{f}+1\right)I+L\right]C\varepsilon_{1}+\Gamma \left(I+L\right)\varepsilon_{2}+\Gamma \left(L_{f}I+L\right)C\varepsilon_{3},{\left\|\Delta u_{k+1}\left(t\right)\right\|}_{\lambda }\leq \left\|I-\Gamma CB\right\|{\left\|\Delta u_{k}\left(t\right)\right\|}_{\lambda }+\Gamma \left(L_{f}I+L\right)CB{\left\|h\left(t\right)\right\|}_{\lambda }+\varepsilon \varepsilon =e^{-\lambda \left(t-\theta \right)}\left[\Gamma \left[\left(L_{f}+1\right)I+L\right]C\varepsilon_{1}+\Gamma \left(I+L\right)\varepsilon_{2}+\Gamma \left(L_{f}I+L\right)C\varepsilon_{3}\right],{\left\|h\left(t\right)\right\|}_{\lambda }\leq \frac{1-e^{\left(L_{f}-\lambda \right)T}}{\lambda -L_{f}}{\left\|\Delta u_{k}\left(t\right)\right\|}_{\lambda },{\left\|\Delta u_{k+1}\left(t\right)\right\|}_{\lambda }\leq \left[\left\|I-\Gamma CB\right\|+\frac{1-e^{\left(L_{f}-\lambda \right)T}}{\lambda -L_{f}}\Gamma \left(L_{f}I+L\right)CB\right]{\left\|\Delta u_{k}\left(t\right)\right\|}_{\lambda }+\varepsilon ,\lim_{k\to \infty }{\left\|\Delta u_{k}\left(t\right)\right\|}_{\lambda }\leq \frac{\varepsilon }{1-\alpha },\lim_{k\to \infty }\underset{t\in \left[0,T\right]}{sup}\left\|\Delta u_{k}\left(t\right)\right\|\leq \frac{\varepsilon e^{\lambda t}}{1-\alpha },\left\|\Delta x_{k}\left(t+\theta \right)\right\|\leq B\overset{t-\theta }{\underset{-\theta }{\int }}e^{L_{f}\left(t-\tau \right)}\left\|\Delta u_{k}\left(\tau \right)\right\|d\tau +\varepsilon_{1}+\varepsilon_{3},{\left\|\Delta x_{k}\left(t+\theta \right)\right\|}_{\lambda }\leq B{\left\|h\left(t\right)\right\|}_{\lambda }+e^{-\lambda \left(t-\theta \right)}\left(\varepsilon_{1}+\varepsilon_{3}\right),{\left\|\Delta x_{k}\left(t+\theta \right)\right\|}_{\lambda }\leq \frac{1-e^{\left(L_{f}-\lambda \right)T}}{\lambda -L_{f}}B{\left\|\Delta u_{k}\left(t\right)\right\|}_{\lambda }+\varepsilon ,\lim_{k\to \infty }{\left\|\Delta x_{k}\left(t+\theta \right)\right\|}_{\lambda }\leq \beta +\varepsilon ,\lim_{k\to \infty }\underset{t\in \left[0,T\right]}{sup}\left\|\Delta x_{k}\left(t\right)\right\|\leq e^{\lambda t}\left(\beta +\varepsilon \right),\left\|\Delta y_{k}\left(t+\theta \right)\right\|\leq C\left\|\Delta x_{k}\left(t+\theta \right)\right\|+\varepsilon_{2},\lim_{k\to \infty }{\left\|\Delta y_{k}\left(t+\theta \right)\right\|}_{\lambda }\leq \left(\beta +\varepsilon \right)C+e^{-\lambda \left(t-\theta \right)}\varepsilon_{2},\lim_{k\to \infty }\underset{t\in \left[0,T\right]}{sup}\left\|\Delta y_{k}\left(t\right)\right\|\leq e^{\lambda t}\left(\beta +\varepsilon \right)C+e^{\lambda \theta }\varepsilon_{2}. \end{array}$$

After the optimized function design is determined, its maturity is evaluated to improve the design process. According to the ILCS design of smart products, the evaluation index of the optimization function is summarized as the smart product working model and the degree to which ILCS simulates the actual working conditions of smart products [13]. The operating system of smart products is almost nonlinear, often with time lag, interference, and arbitrary initial states. The closer the working model is to the actual situation, the more reliable the optimization. Orbital optimization algorithm: convergence is a prerequisite for measuring the success of the ILC algorithm. Only when the ILC algorithm converges, the actual output of the smart product can reach the best solution. The best solution is obtained with a certain precision to achieve the goal of optimization. System robustness: tracking system performance under various interferences [14]. When interference exists, the output of the iterative learning controller can converge to the neighborhood of the desired trajectory; after the interference disappears, the actual output of the system converges to the target trajectory. The evaluation criteria are high optimization accuracy, high reliability, and short response time. Similarly, the use of triangular fuzzy numbers to evaluate the maturity of the optimization function and the evaluation process, see the following. When analyzing the evaluation results, the undesirable optimization function design should be improved. To ensure the realization of the improved optimization function, the ticketing cost and customer value must also be considered.

### 3.2. Design Method of Autonomous Function

Autonomy is the last function of smart products, which is realized by ANFIS and multiagent systems. ANFIS processes information from monitoring, control, and optimization functions, and passes the processed information to multiple ANFIS systems [15]. The multiagent system carries out information distribution, uses knowledge base and Q-learning algorithm for decision-making analysis, and realizes autonomous functions. The fuzzy number of triangles evaluates the maturity of autonomous functions and improves the design of autonomous functions. The information from the monitoring, control, and optimization functions needs to be processed first. This is a process of multiple inputs and outputs.

(5) $$\begin{array}{c} \begin{array}{c} R=A\times B\times C\to D\\ =\left\{\left[A_{1}\times B_{1}\times C_{1}\to D_{1}\right],\left[A_{2}\times B_{2}\times C_{2}\to D_{2}\right],\ldots ,\left[A_{m}\times B_{m}\times C_{m}\to D_{m}\right]\right\}\text{.} \end{array} \end{array}$$

Here, according to the formula, *a* is monitoring information, *b* is control information, and *c* is optimization information. The rule base contains *m* rules, and each rule exists in the form of multiple inputs and a single output. Since the *m* rules are independent of each other, the MIMO process can be decomposed into *m* MIMO processes. The design process of autonomous functions of smart products is shown in Figure 1.

Taking into account the advantages of autonomous learning of neural networks and fuzzy inference of fuzzy systems, ANFIS uses the back propagation algorithm or a hybrid algorithm of the back propagation algorithm and least square method to learn input and output data pairs, and obtain fuzzy membership functions and fuzzy rules independently so that the constructed fuzzy inference system (such as the Takagi-Sugeno model) can better simulate the actual input-output relationship. The learning process calculates the error between the actual output value and the target value and adjusts the system parameters through error back propagation until the system error is met. Therefore, ANFIS is used to solve the multiinput problem of autonomous functions (as shown in Figure 2).

In the first layer, the input information blurs the output function of node *i*, shown as follows:

(6) $$\begin{array}{c} O_{i}^{1}=\mu_{A_{i}}\left(x\right),O_{i}^{1}=\mu_{B_{i}}\left(y\right),O_{i}^{1}=\mu_{C_{i}}\left(z\right)\text{.} \end{array}$$

Here, *x y* and *z* are input monitoring control and optimization information, *A*_*i*_, *B*_*i*_, and *C*_*i*_ are fuzzy sets of monitoring control and optimization, and 1 is the member shiv function value of *A*_*i*_, *B*_*i*_, and *C*_*i*_. In other words, the order in which *x*, *y,* and *z* belong to *A*_*i*_, *B*_*i*_, and *C*_*i*_ is a subordinate function, and this order is usually chosen so that the maximum value of the Gaussian or Bell function is 1 and the minimum value is 0. Take “Smart Scanning Robot” as an example. In the second layer, the input signal multiplication method multiplies the input signal to calculate the reliability of the rule.

(7) $$\begin{array}{c} \omega_{i}=\mu_{A_{i}}\left(x\right)\times \mu_{B_{i}}\left(y\right)\times \mu_{C_{i}}\left(z\right)\text{,}\\ \varpi_{i}=\frac{\omega_{i}}{\sum_{i=1}^{m}\omega_{i}}\text{,}\\ O_{i}^{4}=\varpi_{i}f_{i}=\varpi_{i}\left(p_{i}x+q_{i}y+t_{i}z+r_{i}\right),\\ O^{5}=\sum_{i=1}^{m}\varpi_{i}f_{i}=\frac{\sum_{i=1}^{m}\omega_{i}f_{i}}{\sum_{i=1}^{m}\omega_{i}}. \end{array}$$

### 3.3. Design Principles of Modular Furniture

The powerful functions and important advantages of modular furniture are obvious to everyone, but its design is not a direct and rough decomposition and functional transplantation of traditional furniture. Not all types of modular furniture are suitable for small- and medium-sized comprehensive bookstores. Modular furniture has many models and there are countless variations. When designing, there are actually rules to follow for basic modules and combinations that seem to have no rules.

The golden ratio, ergonomics, etc. may also affect the spiritual needs of users and the creation of the space atmosphere. However, with the diversification of small and medium-scale integrated bookstore space development, the design standard is not just the comfort of modular furniture. The seemingly applicable standards require flexibility to make each piece of furniture more scientific and reasonable within its own functional scope. For example, when considering the width of a standing reading shelf, the baffle is placed at a lateral distance of 45°, which not only ensures comfort but also emphasizes space saving; for example, compared with the table in the restaurant area, the reading table is slightly smaller than the standard value Wider, you can put more books, use distance to hinder communication, you can better create a quiet reading and self-thinking environment. The desktop size of the dining area should be narrow and standard to shorten the distance. This is the scientific, reasonable, and flexible design principle of as many “ergonomics” as possible for the so-called multifunctional area.

If you compare modular furniture to “mosaic,” it may be the most appropriate. Each basic element has its own characteristics, single but abstract. However, when several elements are continuously combined, people will gradually realize its overall meaning. Therefore, the design of modular furniture for bookstores must consider the independence of the individual and follow the principle of the overall application. In general, the following points should be considered for overall applicability: (1) “multiple births” effect. Since the uniform appearance is the most direct and complete, the color, material, and contour type of the module combination must be consistent. It is recommended to keep the same state after free change and reversal; (2) the versatility and interchangeability of the module. When the combination of modules does not have a fixed pattern or any module can be replaced, it fully reflects the overall combination's adaptability to location and individual, so a universal connection method must be used in the design; (3) the continuity of module combination. The most amazing performance of modular furniture is whether there is any mutual generation. To better adapt to spaces of different sizes, it must have a certain continuity to have an overall concept.

Even small- and medium-sized bookstores, there is not very few furniture in the space. In addition to later consumption and maintenance, it is not advisable to pay attention to one thing and lose the other. We must follow the design principles of saving and material recycling. To achieve high output and low consumption, we can start from two aspects: high output of furniture manufacturing and low consumption of furniture use. The intervention of modular design means mass production, and its versatility also minimizes maintenance and replacement costs. In the design process, the module design is tried to be made close to the raw material itself to reduce the difficulty of the manufacturing process. In manufacturing engineering, a reasonable selection of materials is made. Only economy and materials can form a smooth circulation system, and spiritual culture can be better inherited.

The original intention of modular furniture is to provide people with more comfortable and humanized services rather than turning a beautiful and comfortable space into a Torah. IKEA modular furniture has always been loved by people all over the world, but no matter how affordable and applicable, due to uneven stress, it results in the death of children and people are far away from it. In particular, small- and medium-sized comprehensive bookstores have the characteristics of publicity and openness. In the face of a variety of audiences, we should pay attention to prevention, especially the protruding or sharp outline of the surface of furniture products; there are unfixed and falling modules in the furniture system; the furniture is folded because the mechanical performance of the products is not up to standard or the bearing capacity is overloaded or the manufacturing materials produce harmful substances. In a word, no matter how easy the shape and function of furniture are to change, there is no doubt that the principle of safety design is strictly followed.

Furniture and people have a close “skin blind date” relationship. Good furniture can not only bring people a comfortable feeling but also protect or improve the physiological function of the human body in the long-term process and ensure the emotional health of users. This good effect is reflected in the scale and shape of the furniture, which is based on the design principles of ergonomics. According to the size and range of activities of age and gender and the use of different furniture functions and other needs, the size of the furniture itself has to be restricted and the distance between furniture and furniture has to be standardized to ensure the needs of the different number of users. As modular furniture is made of splicing modules, according to the size of the overall furniture, different users have different functions for furniture size.

## 4. Modular Furniture System Design Based on Wireless Sensors

### 4.1. System Design Overview

The smart home wireless control system is mainly based on the smart home system software iotv2 CC2530 hardware system and can control the home equipment of a single user. The system consists of a central server, a smart phone, and a personal computer with a wireless sensor network for centralized management and control of the entire building. All the information collected by the sensor nodes is stored in the real-time server database. Android phones, PDAs, and tablets are gateways, and the server transmits the server through the gateway through the Ethernet on the network (4 G/3 G/Internet/GPRS, etc.) through the CC2530 system. To realize the remote control function of home equipment, the system eliminates the complexity of hardware controller design, does not need to destroy the room layout, does not need to buy new electrical appliances, is simple to install, and saves user costs. The system can not only connect lighting equipment and general equipment, it can also be connected to other equipment, adapt to the needs of new smart life, and has a high degree of scalability. The overall design of the smart home system is shown in Figure 3.

The central server is the main controller of the entire smart home system, controlling all home appliances, including televisions and lighting equipment. The control commands of lighting appliances, infrared household appliances, and various sensors are stored here. Through the alternate interface of the control center, the temperature sensor is equipped with sensors of the intelligent control system, which realizes the convenience of household equipment. The sensors in the system include temperature sensors, smoke sensors, and light intensity sensors. These sensors are connected to the subcontroller (2.4 G module) through a specific circuit module according to their working characteristics. The system collects and analyzes the operating status information of the equipment in real-time. If an abnormality occurs, the status information and abnormal analysis result will be sent to the control center and an alarm will be issued with a “beep”. In this way, the user can know what happened in a short time and react first. The design of the smart home system is divided into two parts: software design and hardware selection. The software mainly includes the design of Android applications, the design of the control system under the Bash architecture, and the communication protocol between wireless sensor nodes, that is, the 2.4 G module design.

### 4.2. System Hardware Selection

Smart home 2.4 G wireless control system uses tiiotv2-2530 hardware platform, a smart gateway, and some subnodes can be configured with three detailed node modules, power module board sensor control module, and a wireless node module. There are mainly three wireless node modules. Module configuration, high-frequency carrier microcontroller wireless communication module, and 2.4 g frequency antenna power module board: power transmission to the system, connection between wireless node module and sensor control module, main power mode can drive battery power or reserve power external DC power supply interface. Sensing and control module: users can also expand their sensor and controller units through the bus. The whole module is a 5VDC power input, built-in DC/DC chip. The input 5VDC power requires 3.3 V and the maximum output current is 200 mA. The single-chip solution used in this system is used in the 2530 system planning stage by extracting the chip signal at the module level and + manual reset chip and reliable phase reset is performed. The 2-wire debugging interface (hardware option operation) is started through the dedicated 5-pin FPC socket. To convert it to a standard debugging plug, an additional expansion board is required. The wireless node module uses two side-by-side 20-pin sockets to send and receive signals. Pin socket 1 pin definition is as shown in Table 1. Pin socket 2 pin definition is as shown in Table 2.

All sensors and controller modules operate uniformly under the control of the 2530 module and have the same control interface, including control signals and physical dimensions. The sensor module uses two rows of 20-pin sockets supported by the power board to communicate with the wireless node module, which is controlled by the wireless node module. The module types supported by the system are introduced as shown in Table 3.

The chip uses EEPROM to complete the ID design and storage of all modules, the interface is IIC, the module characteristic attribute is 2 bytes, the address is 0 and 1, the first byte is used to describe the working mode and attributes, and the second byte is used to describe specific equipment. After he code 2530 is turned on, the current valid ID code of the sensor module or controller module is read from the EEPROM, and the subsequent boot process is determined according to the ID code, mainly the configuration of the IO port and the functional module. The front-end hardware part is composed of cameras and video compression chips. The camera uses a JVCCCD camera, and this design uses a CDD camera. The video compression chip is designed based on TI's DaVincTM series of high-resolution processors tms320dm365. The processor continues the DaVincTM series DM355 processor architecture and integrates the H.264 high-resolution codec processor MJCP, which supports the ARM926EJ-S core and the H.264/MPEG-4 high-resolution video codec together. The data are collected by the camera and controlled by functions such as ARM926EJ-S, H.264 encoding, dual-stream control, and data storage. Finally, it is output through the digital RGB/YUV interface.

### 4.3. Software System Design

The smart home control system uses two software architectures: B/S and C/S. The browser client can access the remote server through wired or wireless Internet (hammer mode), and the Android client application can access the remote server wirelessly. B/S (Browser/Server) is a software architecture improved and developed under the C/S mode. Users mainly implement related functions through the browser and the server is mainly used to implement the logic of things. Compared with the traditional C/S model, the B/S-based software structure not only reduces the load on the client but also reduces the difficulty of future use and maintenance and reduces the cost of use. There are many ways to use the B/S architecture to access the remote database (LAN/WAN/Internet). The advantages of B/S architecture, especially the emergence of cross-platform languages (JAVA), emphasize the advantages of B/S architecture. The system can implement the control system of the text more quickly and effectively. The central control module is wirelessly connected to the indoor subnodes to realize the orderly exchange and management of home appliance data. The data retrieval server is the core of the entire control system, the central node of information management, and the bridge between the client and the management device. The client manages all the data received from the client's control room in an upward and downward manner and the control and management of all the corresponding equipment received by the client up and down realize that the remote server is actually optimized management software. Display the operating status and parameters of on-site electrical equipment and remotely control the equipment. The system architecture is shown in Figure 4.

The Android-based control system uses a simple Android interactive graphical interface. Not only is it easy to use, but it is also highly convenient and can be operated anytime, anywhere. The system includes six detailed modules: scene, monitoring, function, area, and system. The functions of the program mainly include high-sensitivity signal monitoring, electrical equipment switch control, infrared human body monitoring, emergency alarms, etc. It is very convenient for abandoned children, the elderly, and company employees.

### 4.4. System Implementation Based on Wireless Sensors

To make the smart home control system run stably, it is necessary to design the system according to the SimpliciTI protocol to make it suitable for the home environment.  Table 4 shows the detailed description of each data in the frame format.

The specific architecture of the intelligent system is shown in Figure 5. The presentation layer can express the content after transcoding, which is the interactive page presented to users by the system at last. This layer is divided into two modules: the view layer and the control layer. The former is used to display the interface for users to operate, while the latter is used to verify, store, and control the page skipping of data submitted by users. For users, the presentation layer is a mini program running on the browser. In fact, the network socket video frequency monitoring function was also implemented in this way. Control layer: as the core layer of the system, the control layer plays the most important role and the largest task, including providing external services such as video server, web server, and peripheral control program. Data layer: a large amount of information generated during the whole system operation is saved in the call through this layer. The main data saved and called are XML files of tables in database and file system.  Figure 6 shows the system structure.

A device refers to one that communicates with an external device in accordance with a prescribed protocol. The interface includes serial ports, Ethernet, USB, etc., but the final connection to the Internet of Things service is Ethernet. If the device is a non-Ethernet interface, the corresponding adapter must be converted to a network interface. For example, in a wireless sensor network application, the coordinator is the device. But the output is serial data, which needs to be connected to the Internet of Things service through a “serial network port” converter. The communication between the device and the Internet of Things service must be in accordance with the prescribed protocol and process. The device communication process is divided into two stages. The first step is to communicate with the intermediate service. The device mainly establishes a connection with the intermediate service to complete the initialization of the device type identification and certain communication parameters. After the first stage is completed it enters the second stage. The second phase requires the cooperation of high-level applications. If the upper-layer application is also connected to the service, the device starts to communicate with the upper-layer application through the service. At this time, the role played by the service is data forwarding. The communication between the upper-level application and the device without processing data is coordinated.

## 5. Analysis of the Modular Furniture Design Strategy

### 5.1. The Design Method of Modular Furniture

Compared with ordinary traditional furniture, the characteristics of modular furniture are eye-catching. Regardless of form or function, modular furniture has broken through traditional boundaries, giving furniture more meaning. This means that the design of modular furniture is also different from traditional furniture, and not only the overall combination form must be considered, but also the establishment of single units. In addition, the specific environment of the small and medium comprehensive bookstore also has a certain impact on its design techniques. The form and function of modular furniture are closely related with the combination of modules. It is precisely because of the diversity of combinations that modular furniture can be “variety.” (1) As the name implies, the package layout and combination design select the module with the largest volume as the outer frame, and other modules can be classified into the largest module according to the order of size. This design method can make the furniture module an individual, meet the needs of multiple people at the same time, and free up more space for use without the need to combine or accept. Due to the characteristics of module combination and splitting, it can be based on the acceptance object. The appropriate module for the size is chosen and the internal space is effectively used. (2) Stackable type is also called building block type. Like building blocks, modules are furniture stacked according to the needs of users. To improve the safety of the furniture, some stackable furniture modules will adopt a fixed connection structure to ensure that the furniture will not collapse under the action of external forces. This design method is simple and convenient to operate, can quickly and effectively decompose scattered furniture into parts, and clean and organize the environmental space. (3) The method of assembly design is similar to the method of building blocks, but the modules are fixed to each other through connectors such as screws and bolts or the grooves and structures of the modules themselves. By connecting components and connecting structures to assemble modules, various shapes of furniture can be made, which are very flexible. (4) The splicing type divides the modular furniture into the furniture type with connecting pieces and plates as the assembly parts, namely the panel furniture, which is the most widely used and most complete type of modular furniture. Various styles of furniture can be combined according to the size of the board and the shape of the connecting piece.

The main market competitiveness of modular furniture is its versatility. However, as one of the important decorations of bookstores, the “look” of furniture cannot be ignored. In addition to considering the powerful functions of the module combination, the design must also follow the rules of formal beauty, such as the color, material, and shape of the furniture. This combination of art and function makes modular furniture one of the characteristics of bookstores and can attract customers who experience consumption. The design method of integrating art into functions is not only oriented to a single module but also simulates the combined overall furniture, ensuring that no matter how the user is reorganized consistently, the bookstore environment can bring in people a sense of fun.

Furniture design in bookstores affects creativity in many ways. In the method of integrating the experience into bookstores, modular furniture plays an important role. (1) The overall design of furniture is one of the elements that change the atmosphere of the space. The so-called “successful furniture, failed furniture”, if the design of furniture only pays attention to the form and function of the individual, and does not pay attention to the overall coordination of the space, it will be exactly. On the contrary, it will deteriorate the atmosphere of the space and even hinder the use of certain functions. (2) As a furniture system, modular furniture should not only protect the independence of each module but also consider the integrity of the combination; as a space element, modular furniture should not only provide comprehensive functions but also pay attention to the overall coordination of the space. Only by focusing on the overall development of each link can a good experience space environment be created. (3) Interesting furniture design text has the magical power to make people feel on the scene, while modular furniture can truly make people live in the world of children.

### 5.2. Development Trend of Modular Furniture

Modular furniture has gradually entered people's daily lives. With the increasing demand for cosmic experience and the popularization of technological intelligence, the design of modular furniture has become more humane, and the scope of application will also expand. With continuous maturation and development of the society and economy, people's needs are increasing day by day, and the optimization and progress in the design and application of modular furniture are constantly promoted. Designers must always pay attention to the development of science and technology and the changes in human needs. The modularization of modular furniture is more reasonable, the function is more complete, the shape is more changeable, and the connection method is more scientific. Therefore, some bold predictions can be made.

The main contents are as follows: (1) in the progress and development process of modern artificial intelligence in the continuous acceleration and in the application of modular furniture, artificial intelligence terminal system has become an indispensable part. In the future, the embedding and development of artificial intelligence devices have emerged in the production and research and development process of furniture, which can not only provide the basic efficiency of furniture but also enhance the interaction between people and furniture to provide personalized services for people's emotional and psychological needs. In addition, artificial intelligence transplantation can provide uninterrupted humanized services, save human resources, and conform to the design principles of sustainable development. (2) With the development of modular automation, self-transforming DIY models are not limited to material changes that directly contact the human body and the manufacturing process, not just artificial parts. According to the combination of mobile terminal and furniture, the components of modular furniture in the future may apply the principle of automation. Through the intelligent design of computer calculation, the automatic module components are automatically deformed to form new furniture. (3) The reproducible mass production of modular furniture for parametric production development is its biggest feature. The premise of this mass production is that this series of modules can be well applied to different collars and have a high degree of matching with other parts. Therefore, calculating the relevant matching value of the module components is an important link that needs to be considered in the design process and requires a lot of time and effort. Relevant data from the parameter library are collected, the computer terminal is used to analyze the relationship between various data, the combination rule is found, and these parameters are used to configure the intelligent module. To improve the comfort of modular furniture, we provide scientific and reasonable division and combination of furniture modules. I think that with the continuous advancement of science and technology, people have put forward more advanced design concepts and design methods, and the development potential of modular furniture will also be greater. Big digging has the characteristics of fast production speed, large output, and multiple functions, and has good applications in the space environment of the data age.

## 6. Conclusion

Based on people's actual life needs, this paper designs an intelligent system with Android system as the server, which can run indoors and interact with people. According to the previous research results of this system, the relevant literature is analyzed and sorted out as well as the special research and the development status and future development trend of the internal software of smart phones are deeply discussed. Android's smartphone interior management system designed a plan. Finally, the software design of the Android client is completed under the Eclipse development tool. The smart home control system designed in this paper supports data monitoring, processing, storage, and other functions of the home environment. Module functions include electrical equipment control, high-sensitivity signal monitoring, remote intelligent anti-theft system, etc., which fully meet the needs of most families. This framework is based on customer needs and aims to monitor, control, optimize smart products and realize autonomous functions. The content of the framework includes the determination and analysis of requirements based on the maximization of customer value, the conversion of customer requirements into technical attributes, the design of optimization and independent functions, and the design process and key technologies that support the realization of the content of the framework.

## Figures and Tables

**Figure 1:** Design process of autonomous functions of smart products.

**Figure 2:** ANFIS structure of smart products.

**Figure 3:** Smart home overall design structure.

**Figure 4:** System architecture.

**Figure 5:** The architecture of the system.

**Figure 6:** System structure.

**Table 1:** Pin socket 1 pin definition.

Serial number	Name	Type	Detailed description
1	VCC	PWR	3.3 V power input pin
2	VCC	PWR	3.3 V power input pin
3	BDECT	I	Use type detection input, power board = *L*; smart motherboard = *H*
4	RSV2	P	Reserved pins, do not connect
5	RS V0	P	Reserved pins, interconnected with corresponding positions on the sensor board
6	RSVI	P	Reserved pins, interconnected with corresponding positions on the sensor board
7	JTAG_VCC	PWR	JTAG debug interface power pin
8	JTDO	0	JTAG debugging interface TCK. pin (2530 chip P2_l pin)
9	JTCK	I	JTAG debug interface TCK pin (P2_2 pin of 2530 chip)
10	JTMS	I	JTAG debug interface TMS pin
11	JTDI	0	JTAG debug interface TDL pin
12	JTRST	I	JTAG debug interface JTRST pin
13	GND	PWR	GND pin of 3.3 V power supply
14	GND	PWR	GND pin of 3.3 V power supply
15	LCD_AO	0	AO control bit of LCD controller
16	LCD_SCL	0	SCL control bit of LCD controller
17	LCD_SDA	IO	SDA control bit of LCD controller
18	LCD-CS	0	CS control bit of LCD controller
19	LCD_RESET	0	RESET control bit of LCD controller
20	RESET	I	Module overall reset control signal input, low effective

**Table 2:** Pin socket 2 pin definition.

Serial number	Name	Type	Detailed description
1	VCC	PWR	5 V power input pin
2	VCC	PWR	5 V power input pin
3	ADIN0	ADINO	Analog input pin, AD acquisition input 0
4	ADIN1	ADIN1	Analog input pin, AD acquisition input 0
5	GND	GND	GND pin of 5 V power supply
6	GND	GND	GND pin of 5 V power supply
7	ESCL	0	SCL pin of expansion device IIC bus
8	ESDA	IO	The SDA pin of the expansion device IIC bus
9	ETXD	0	TXD pin of UART, TTL level
10	ETXD	I	RXD pin of UART, TTL level
11	EGPI00	IO	External logic input pins, used as networking control buttons when the system is started
12	EGPI01	IO	External logic input pins, used as networking control buttons when the system is started
13	GND	PWD	GND pin of 5 V power supply
14	GND	PWD	GND pin of 5 V power supply
15	EG POO	0	External logic control output pin, programmable control
16	INT	I	External logic control output pin, programmable control
17	EREQ	0	Peripheral function request handshake request signal output
18	EACK	I	Peripheral function request handshake response signal input
19	RSV5	P	Reserved pins, do not connect
20	RESET	I	Module overall control signal input, low effective

**Table 3:** Module function introduction.

Serial number	Name	Function introduction
1	Current sensor	The measurement range is 0.5 A ∼ 2 A, the resolution is 0.01 A, at least the ad of lobit is used.
2	Temperature and humidity sensor	The temperature measurement range is −20°C ∼ i30c, and the measurement accuracy is 0.1°C; the humidity measurement range is 0–100%, and the accuracy is 0.1%.
3	Illumination sensor	It is realized by one channel ad, and the measurement range is. The resolution is 101x.
4	Infrared control output	Using serial port + CPU scheme, three groups of IR are output.
5	Relay control	Using IIC extended GPIO chip, 4 groups of relays, normally open/normally closed, can be configured arbitrarily.

**Table 4:** Detailed description of each data in the frame format.

Name	Length (bit)	Value	Description
Message type	8	01	Electrical control (control center one electrical equipment module)
		02	Temperature and humidity control (control center a temperature and humidity module)
		03	Temperature collection (temperature control module-control center)
		04	Infrared learning (an infrared control module in the control center)
		05	Infrared transmission (infrared centralized module one control center)
		06	Infrared control (an infrared control module in the control center)
Destination address	8	0–255	The address of the device receiving the control command
Source address	8	0–255	The address of the device sending the data
Data length	8	0	No data
		1–255	Actual number length
Valid data	n		The actual data

## Data Availability

The data used to support the findings of this study are available from the author upon request.
